# The epidemiology, clinical presentation, and predictors of severe Tick-borne encephalitis in Lithuania, a highly endemic country: A retrospective study of 1040 patients

**DOI:** 10.1371/journal.pone.0241587

**Published:** 2020-11-19

**Authors:** Daiva Radzišauskienė, Jurgita Urbonienė, Gintaras Kaubrys, Saulius Andruškevičius, Dalius Jatužis, Elžbieta Matulytė, Karolina Žvirblytė-Skrebutienė

**Affiliations:** 1 Clinic of Infectious Diseases and Dermatovenerology, Institute of Clinical Medicine, Faculty of Medicine, Vilnius University, Vilnius, Lithuania; 2 Center of Infectious Diseases, Vilnius University, Vilnius, Lithuania; 3 Clinic of Neurology and Neurosurgery, Institute of Clinical Medicine, Faculty of Medicine, Vilnius University, Vilnius, Lithuania; Hospital Dr. Rafael A. Calderón Guardia, CCSS, COSTA RICA

## Abstract

**Introduction:**

In recent decades, the incidence of Tick-borne encephalitis (TBE) has been increasing and posing a growing health problem because of the high costs to the healthcare system and society. The clinical manifestations are well studied but there is a lack of research analyzing the severity of the disease.

**Objective:**

The aim of this study was to analyze the epidemiology and clinical presentation of severe TBE, to identify the predictors for a severe disease course, and also predictors for meningoencephalomyelitic and severe meningoencephalitic/encephalitic forms.

**Methods:**

A retrospective study was conducted in the Center of Infectious Diseases and the Center of Neurology at Vilnius University Hospital Santaros Klinikos in the years 2005–2017 to describe the clinical and epidemiological features of TBE in adults.

**Results:**

1040 patients were included in the study. A total of 152/1040 (14.6%) patients had a severe course. The highest proportion of severe cases, reaching 41.2%, was reported in the 70–79 year-old age group. A total of 36/152 (23.7%) severe patients presented meningoencephalomyelitis. Myelitic patients were older, were frequently infected in their living areas, and usually reported a monophasic disease course compared with severe meningoencephalitic/encephalitic patients. Severe meningoencephalitic/encephalitic patients, compared with non-severe meningoencephalitic/encephalitic, were older, less often noticed the tick bite, and often had a monophasic course. The sequelae on discharge were observed in 810/1000 (81%) of patients.

**Conclusions:**

The prognostic factors associated with a severe disease course and severe meningoencephalitic form are: older age, comorbidities, a monophasic course, a fever of 40˚C and above, CRP more than 30 mg/l, CSF protein more than 1 g/l, delayed immune response of TBEV IgG, pathological findings in CT. Age above 60 years, presence of CNS disease, bulbar syndrome, pleocytosis 500x10^6^/l and above, and delayed immune response of TBEV IgG are predictors of the most severe myelitic form.

## Introduction

The Tick-borne encephalitis virus (TBEV) causes a serious infection of the central nervous system (CNS). This is the most frequent viral CNS infection in endemic areas [1, 2]. During the last few decades, the incidence of TBE has been increasing and posing a growing health problem because of the high costs to the healthcare system and society [2–5]. TBEV has its natural foci where it circulates among its vectors, ticks and reservoir hosts such as rodents and small mammals. According to Ecker, TBEV consists of 3 subtypes: European (TBEV-EU), Siberian (TBEV-Sib), and Far East (TBEV-FE) [6]. Russian virologists have claimed 2 new subtypes, strain 178–19 and strain 886–84, both isolated in the Lake Baikal region in Siberia [7]. In Europe, TBEV-EU circulates in the Baltic countries, and in parts of Finland, TBEV-Sib and TBEV-FE subtypes virus strains have been isolated. TBEV-Sib subtype is the most common and has been found almost everywhere in TBEV endemic areas.

Although the disease is preventable by vaccination, several thousand people fall ill with TBE each year [8]. In Europe and Asia, between 10 000 and 15 000 cases are reported annually [4, 9]. The majority of patients infected with TBEV-EU present a biphasic course. The most frequent symptoms are fever and headaches. The course of TBE is classified as mild, moderate, and severe, depending on the affected parts of the CNS. Severe forms of TBE progress to loss of consciousness, flaccid paralysis of the extremities involving the respiratory muscles, and even death. The clinical manifestation of the disease is well studied [4, 10–12], but there is a lack of studies analyzing the severity of the disease. In literature, there have been few studies analyzing the prognostic factors of severe meningoencephalomyelitis (myelitis) and severe meningoencephalitis (ME) [13, 14].

The aim of this study was to analyze the epidemiology and clinical presentation of severe TBE, and to identify the predictors of the severe course of the disease, and also predictors for meningoencephalomyelitic and severe meningoencephalitic/encephalitic forms.

## Methods

### Patients and study design

A retrospective study was carried out to describe the clinical and epidemiological features of TBE in adults. The study took place at the Center of Infectious Diseases and the Center of Neurology of Vilnius University Hospital Santaros Klinikos in 2005–2017. These are referral centers for adult infectious diseases and nervous system diseases in eastern Lithuania. They serve a population of 809 000, which is 27% of the country’s population.

Cases were defined based on laboratory results and precisely documented clinical characteristics. The clinical criterion was a person with signs of CNS inflammation. The laboratory criteria were the presence of specific TBE immunoglobulins (IgM and IgG) in serum, or proven intrathecal synthesis of TBE IgM. The diagnosis of patients without cerebrospinal fluid (CSF) investigation (n = 40/1040(3.8%)) was based on clinical presentation, seroconversion of TBV IgM and IgG, and exclusion of other diseases. The inclusion criterion was all patients 18 years and older diagnosed with TBE. The exclusion criteria were patients vaccinated against yellow fever and Japanese encephalitis and/or patients infected with other *flaviviruses*. Confirmed cases were included for further analysis. EpiData (v.3.1: The EpiData Association, Odense, Denmark) was used for data entry and data documentation. The variables included demographic data, comorbidities, the date of illness onset, the duration of hospitalization, the symptoms, signs, and duration of the 1st and 2nd phase of infection, blood tests, CSF tests, the data of computed tomography (CT), and electromyography (EMG). Epidemiological data such as the date and the geographical areas of tick bites, consumption of unpasteurized milk or milk products, vaccination against TBE and other *flaviviruses* and traveling in *flavivirus* endemic areas, were collected.

### Laboratory diagnosis

TBE was laboratory tested by the demonstration of specific IgM and IgG activity in serum or intrathecal specific IgM synthesis by immunological tests of enzyme-linked immunosorbent assay (ELISA). Virion/Serion (Wurzburg, Germany) TBE Virus IgM and IgG (quantitative) kits have been used for detection of antibodies since 2009 (www.virion-serion.com). For test evaluation, the optical density is read by fully automated microplate processor STRATEC GEMINI. For evaluation of antibody concentrations, the processor software uses a lot specific standard curves as well as a lot of specific evaluation tables (included with each test kit). Before testing, samples were diluted with dilution buffer to eliminate rheumatoid factor to avoid false-positive reactions. According to the manufacturer, the sensitivity and specificity of TBEV IgM reaches 99%, the sensitivity of TBEV IgG is 98.9%, and the specificity is 98.3%. EUROIMMUN (Germany) kits were used in years 2005–2008 (www.euroimmun.com). According to the manufacturer, the sensitivity and specificity of TBEV IgM reaches 100% based on INSTAND external quality control data (n = 129).

### Clinical classification

According to clinical presentation, TBE cases were classified into meningitis (M), meningoencephalitis or encephalitis (E) and meningoencephalomyelitis. Patients presenting symptoms and/or signs of parenchymatous disease of the brain such as focal neurological signs, seizures, quantitative and qualitative impairment of consciousness, concomitant with CSF pleocytosis > 5x10^6^/l, were classified as having ME. The diagnosis of myelitis was based on clinical signs of alpha-motor neuron damage: low muscle tone, loss or weakening of reflexes, no pathological reflexes, no pain, no sensory impairment, characteristic development of muscle atrophies, and/or signs of 11th cranial nerve damage, and/or characteristic findings in EMG. Patients with CSF pleocytosis > 5x10^6^/l with lack of symptoms and signs of encephalitis or myelitis were diagnosed as having meningitis. Some patients who had encephalitic symptoms without CSF pleocytosis were classified as having encephalitis.

The course of the disease was classified as severe and non-severe. A severe case was defined as a disease with severe diffuse brain dysfunction: coma, stupor, somnolence for 2 days and more; qualitative altered consciousness if the patient was dangerous to themselves and others with a need for prescription of antipsychotics; and/or at least 3 multifocal CNS signs such as: severe ataxia when patients were unable to walk, severe bulbar syndrome, central paresis, seizures, dysphasia, movement disorders. Patients who presented myelitis were classified as severe.

A fever was defined if the axillary a.m. temperature was 37.3˚C and above or p.m. temperature was 37.8˚C and above [15]. The onset of the illness was defined as the 1st day of fever in the manifestation phase. For 33/1000(3.3%) patients who did not have a fever, the onset of the disease was considered from the occurrence of the 1st neurological sign.

All symptoms and signs present on discharge were classified as mild, moderate, or severe according to the modified Rankin scale. Mild sequelae were those without any impact on the activities of daily life, and patients were able to carry out all the usual duties and activities. Moderate sequelae were defined as residual symptoms or signs that affected activities in daily life, patients required some help and were unable to work in a previous job but were able to walk without assistance. Severe sequelae were those that led to an inability to continue previous activities, unable to walk without assistance.

### Statistical methods and ethics

The statistical calculations were performed using the IBM SPSS version 20.0 for Windows software. Descriptive statistics for categorical variables are presented by absolute and relative frequencies, as for continuous variables, by the mean values, standard deviation (SD), and ranges. The differences between groups were assessed using the χ2 test or Fisher’s exact test. The differences between the means of the continuous variables were tested using the Mann-Whitney test. Univariate and multivariate logistic regression analysis was performed to assess predictors for severe disease course. A *p* value of < 0.05 was considered statistically significant.

The Vilnius Regional Biomedical Research Ethics Committee approved this study in 2014 (No. 158200-14-742-259). A permission to continue the study was granted in 2018 (No. 158200-14-742-PB3-59). The Ethics Committee waived the requirement for informed consent on the basis of the right granted of the Law on Ethics of Biomedical Research of the Republic of Lithuania. The research also obtained a permission from the State Data Security Inspectorate (No 2R-2808 (2.6–1.)).

The confidentiality of the study data is guaranteed. Personal data collected were anonymized and encrypted. No names and no other personal data of the patients were mentioned in the study documents.

## Results

### Epidemiological and demographic data

A total of 1040 patients were included in the study. The mean age was 49.9±16.4 years (min 18 –max 85). A total of 574/1040 (55.2%) patients were men.

The distribution of TBE cases by severity and clinical form is presented in Fig 1. A total of 152/1040 (14.6%) patients had a severe case of illness. The clinical form of the disease was not identified for 40 patients, because lumbar puncture was not performed.

**Fig 1:** Clinical and disease course forms of Tick-borne encephalitis. E–encephalitis, M–meningitis, ME–meningoencephalitis, Myelitis–meningoencephalomyelitis.

The number of hospitalized patients with TBE has been increasing since 2009. The highest number of hospitalized patients was in 2013. The proportion of severe cases varied from 7.1% in 2005 to 26.5% in 2010 (Fig 2).

**Fig 2:** Annual incidence of Tick-borne encephalitis (n = 1040).

The majority of patients with TBE were admitted to hospital in July, August, and September. In 8 out of 13 calendar years, 2 TBE peaks were observed: 1 in July and 1 in early fall (September–October). The highest proportions of severe cases were observed in May, June, and July (Fig 3).

**Fig 3:** Seasonal incidence of Tick-borne encephalitis (n = 1040).

Patients’ basic demographic and epidemiological data are presented in Table 1.

**Table 1:** Epidemiological and demographic data of Tick-borne encephalitis.

Parameters	All patients^ n = 1000	Myelitis n = 36	Severe ME/E n = 116	p_1_	Non-severe ME/E n = 750	p_2_
**Age, years, mean ± SD (min-max)**	49.8±16.4 (18–85)	60.2±15.3 (24–81)	53.7±17.6 (18–85)	0.05	50.0±15.6 (18–85)	0.02
**Male, n (%)**	552 (55.2)	23 (63.9)	63 (54.3)	ns	413 (55.1)	ns
**Inhabitants of cities, n (%)**	599 (59.9)	15 (41.7)	65 (56.0)	ns	456 (60.8)	ns
**History of tick bite, n (%)**	642 (64.2)	23 (63.9)	64 (55.2)	ns	496 (66.1)	0.02
**Milk-borne infection, n (%)**	64 (7.0)	1 (3.2)	8 (8.0)	ns	53 (7.6)	ns
**Infected in living area, n (%)**	359 (46.2)	20 (69.0)	40 (47.6)	0.05	271 (45.6)	ns
**Job-related infection, n (%)**	16 (2.1)	1 (3.2)	4 (4.8)	ns	11 (1.8)	ns
**Incubation period, days, mean ± SD (min-max), n**	11.7±9.9 (<1–61), n = 256	13.3±11.8 (2–29), n = 4	12.4±11.4 (3–49), n = 21	ns	11.6±9.7 (<1–61), n = 207	ns
**Biphasic course, n (%)**	598 (60.0)	10 (27.8)	52 (44.8)	0.07	472 (63.3)	<0.0001
**Duration of 1st stage, days, mean ± SD, (min-max), n**	5.1±3.0 (1–25), n = 467	3.7±2.8 (1–8), n = 4	4.7±3.1 (1–19), n = 39	ns	5.2±3.0 (1–19), n = 369	ns
**Asymptomatic period, days, mean ± SD, (min-max), n**	8.9±5.7 (1–44), n = 458	N.D., n = 0	8.4±5.0 (3–20), n = 39	-	8.9±5.8 (1–44), n = 367	ns
**Pre-existing conditions, n (%)**	433 (43.3)	24 (66.7)	61 (52.6)	ns	323 (43.1)	ns
**CNS disease, n (%)**	27 (2.7)	5 (13.9)	3 (2.6)	0.02	18 (2.4)	ns
Time between hospitalization and fever* onset, days, mean ± SD (min-max), n	5.4±5.6 (-10-57), n = 993	4.0±2.9 (<1–10), n = 36	5.7±6.6 (-4-53), n = 115	ns	5.5±5.7 (-10-57), n = 745	ns

E–encephalitis, ME–meningoencephalitis, p_1_ –myelitis versus severe meningoencephalitis, p_2_ –severe meningoencephalitis versus non-severe meningoencephalitis

^patients with diagnosed clinical form

* 2nd wave of fever if biphasic course, N.D.–not diagnosed, ns–not significant.

Patients with severe TBE were on average 6.2 years older than patients with non-severe TBE (the mean age was 55.3±17.2 vs. 48.8±16.0, p<0.0001). The highest proportion of severe cases, reaching 41.2%, was reported in the 70–79 age group. Myelitic patients were older, were frequently infected in their living area, and more often, although it is statistically not significant, reported a monophasic disease course compared with severe ME/E patients (Table 1).

Severe ME/E patients compared, with non-severe, ME/E patients were older, less often noticed the tick bite, and often had a monophasic course. There was no statistically significant difference in the length of incubation and asymptomatic periods, the duration of 1st stage between groups of myelitic and severe ME/E patients, and between patients with severe and non-severe ME/E.

The most common pre-existing condition was arterial hypertension (n = 254, 25.4%). 6.1% of patients had coronary artery disease, 4.5% diabetes mellitus and 2.7% chronic CNS illnesses. The proportion of comorbidities was higher among severe patients compared with non-severe (85/152 (55.9%) vs. 348/848 (41.0%), p<0.01).

### Clinical presentation

The predominant clinical form of TBE was meningoencephalitis, accounting for 820/1000 (82.0%) of all cases. A total of 36/152 (23.7%) severe patients presented myelitis (Fig 1).

A total of 964/1000 (96.4%) patients presented a mean fever of 39.0 ± 0.7˚C (min 37.3˚C–max 42˚C) with a mean duration of 7.7 ± 5.9 days. The majority of them, 922 (95.6%), had a fever of 38˚C and above. 96.4% (n = 964) of patients complained of headaches at the time of hospitalization. Headaches were less common among severe TBE patients compared with non-severe TBE patients (139/152 (91.5%) vs. 825/848 (97.3%), p<0.0001), and among myelitic patients compared with severe ME/E patients (30/36 (83.3%) vs. 109/116 (94%), p = 0.06).

The most frequent neurological signs were: cerebellar ataxia 819/1000 (81.9%), meningeal signs 617 (61.7%), and extrapyramidal tremor 526 (52.6%). Severe patients presented meningeal signs more often than non-severe, but myelitic patients presented meningeal signs less frequently compared with severe ME/E patients (Fig 4A and 4B). Severe ME/E patients presented parkinsonism less frequently than non-severe ME/E 3/152 (2.6%) vs. 66/750 (8.8%), p = 0.02. There was no statistically significant difference in this sign between myelitic and severe ME/E groups 3/36 (8.3%) vs. 3/116 (2.6%). Non-severe ME/E patients presented extrapyramidal tremor more frequently compared with severe ME/E patients (Fig 4C).

**Fig 4:** Neurological signs of Tick-borne encephalitis. (A) Neurological signs of severe and non-severe TBE. (B) Neurological signs of severe myelitic and severe meningoencephalitic/encephalitic forms of TBE. (C) Neurological signs of severe and non-severe meningoencephalitic/encephalitic forms of TBE. *p<0.05, **p≤0.01, ***p<0.0001.

A total of 202/1000 (20.2%) patients had quantitative impairment of consciousness. Although myelitic patients had this sign less frequently compared with severe ME/E, they were affected more severely (Fig 4B): coma occurred in 12/36 (33.3%) of myelitic patients vs. 3/116 (2.6%) of severe ME/E patients (p<0.0001), and lasted on average 5.3 days longer in myelitic patients compared with severe ME/E patients (6.6±6.3 vs. 1.3±0.6, p<0.05). Consciousness was impaired on the 6th day since the onset of the fever in both groups.

A total of 135/1000 (13.5%) patients had qualitative impaired consciousness and 12 (8.9%) reported hallucinations.

The impairment of cranial nerves was reported in 330/1000 (33%) cases. Severe cases presented a deficit of cranial nerves more often than non-severe (Fig 4). A total of 64/1000 (6.4%) patients presented signs of damage of nuclei of the 3rd, 4th, and 6th cranial nerves. Severe patients developed these signs more often compared with non-severe, as did myelitic patients compared with severe ME/E (25 (16.5%) vs. 39 (4.6%), p<0.0001 and 12 (33.3%) vs. 13 (11.2%), p = 0.002). Myelitic patients presented bulbar syndrome on average 1.9 days earlier compared with severe ME/E patients: accordingly, on 5.5±3.8 (min <1 –max 13) vs. 7.5 ±6 (min<1 –max 23) day since fever onset, p>0.05. The impairment of 7th, 11th, and 12th cranial nerves, and hearing disturbance were rare signs, and were identified respectively in 9/1000 (0.9%), 7 (0.7%), 11 (1.1%), and 21 (2.1%) cases. The 7th cranial nerve was damaged more often in the severe cases group, but there was no statistically significant difference between myelitic and severe ME/E groups. There was no statistically significant difference in hearing disturbance in all groups.

The peripheral nervous system (PNS) was damaged in 48/1000 (4.8%) cases. Myelitic patients presented signs of PNS damage more often compared with severe ME/E 9/36 (25%) vs. 1/116 (0.9%), p<0.0001, but severe ME/E patients had these signs less frequently compared with non-severe ME/E 1/116 (0.9%) vs. 35/750 (4.7%), p = 0.075. 6 out of 9 patients with myelitis and PNS damage had no impaired consciousness. EMG was done for 2 patients and showed fasciculations of proximal muscles of extremities and decreased motor response amplitude. The other 4 patients presented PNS damage 7 days later than myelitic signs.

### Laboratory findings, outcomes and sequelae

Severe cases had more elevated C-reactive protein (CRP), mg/l (15.0±17 vs. 9.6±12.1, p<0.0001), higher pleocytosis (161x10^6^/l ±202 vs. 122x10^6^/l±141, p = 0.07), a higher percentage of neutrophils (34.3±26.6 vs. 21.5±23.9, p<0.0001), a higher level of protein, g/l in CSF (1.0±0.5 vs. 0.8±0.4, p<0.0001), and a higher proportion of pathological findings in CT (n = 11, 20.0% vs. n = 14, 9.7%, p = 0.048) compared with non-severe cases (Table 2). The pathological findings in CT included cerebral edema, intracranial hypertension, and small non-contrast-enhanced hypodensic foci.

**Table 2:** Laboratory findings and outcomes of Tick-borne encephalitis.

Parameters	Severe cases n = 152	Non-severe cases n = 848	p_1_	Myelitis n = 36	Severe ME/E n = 116	p_2_
**Leukocytosis in peripheral blood, cells x10^9^/l**	10.0±3.2	9.7±3.0	ns	9.9±3.1	10.0±3.3	ns
**Neutrophils in peripheral blood, cellsx10^9^**	7.9±3.0	7.2±2.8	0.005	7.8±2.8	7.9±3.0	ns
**CRP, mg/l**	15.0±17	9.6±12.1	<0.0001	14.4±16.8	15.2±17.4	ns
**Pleocytosis, cells in CSFx10^6^/l, mean ± SD (min–max)**	161±202 (0–1306)	122±141 (1–1707)	0.07	246±328 (10–1306)	135±134 (0–645)	ns
**Neutrophils in CSF, %**	34.3±26.6	21.5±23.9	<0.0001	42±29.7	32±25.3	ns
**Protein in CSF, g/l, mean ± SD (min–max)**	1.0±0.5 (0.3–5.8)	0.8±0.4 (0.1–6.2)	<0.0001	1.0±0.3 (0.6–2.0)	0.9±0.6 (0.3–5.8)	ns
**Pathological findings in CT, n (%)**	11 (20.0), n = 55	14 (9.7), n = 145	0.048	3 (23.1), n = 13	8 (19.0), n = 42	ns
**Edema papillae n. optici, n (%)**	9 (9.6), n = 94	27 (6.8), n = 396	0.36	1 (5.9), n = 17	8 (10.4), n = 77	ns
**Length of hospital stay, days, mean ± SD (min–max)**	17.0±13.1 (4–129)	11.0±3.6 (1–41)	<0.0001	26.0±23.1 (6–129)	14.2±6.1 (4–36)	<0.0001
**ICU, n (%)**	125 (82.2)	173 (20.4)	<0.0001	24 (66.7)	100 (86.2)	0.005
**Length of ICU stay, days, mean ± SD (min–max)**	7.0 ±15.0 (<1–127)	2±1.4 (<1–11)	<0.0001	22.0±29.1 (1–127)	3.2±3.2 (<1–26)	<0.0001
**Mechanical ventilation, n (%)**	17 (11.2)	0	<0.0001	13 (36.1)	4 (3.4)	<0.0001
**Sequelae on discharge total, n (%)**	139 (91.4)	671 (79.1)	<0.0001	36 (100)	103 (88.8)	0.04
**Severe sequelae, n (%)**	45 (29.6)	2 (0.2)	<0.0001	33 (91.7)	12 (10.3)	<0.0001
**Deaths during acute period, n (%)**	4 (2.6)	0	0.001	3 (8.3)	1 (0.01)	0.04
**General malaise, n (%)**	100 (67.6)	446 (52.7)	0.001	27 (81.8)	73 (64.0)	0.05
**Headache, n (%)**	26 (17.6)	206 (24.3)	ns	6 (18.2)	20 (17.4)	ns
**Dizziness, n (%)**	45 (30.4)	306 (36.1)	ns	4 (12.1)	41 (35.7)	0.01
**Myalgia, n (%)**	6 (4.1)	12 (1.4)	0.04	2 (6.1)	4 (3.5)	ns
**Radiculopathy, n (%)**	7 (4.7)	15 (1.8)	0.03	6 (18.2)	1 (0.9)	<0.0001
**Cerebellar ataxia, n (%)**	92 (62.2)	409 (48.2)	0.001	19 (57.6)	73 (63.5)	ns
**Extrapyramidal tremor, n (%)**	33 (22.3)	241 (28.4)	ns	8 (24.2)	25 (21.9)	ns
**Parkinsonism, n (%)**	3 (2.0)	51 (6.0)	0.03	1 (3.0)	2 (1.8)	ns
**Impaired respiratory function, n (%)**	6 (4.1)	0	<0.0001	5 (15.2)	1 (0.9)	0.002
**Paresis, n (%)**	37 (25.2)	5 (0.6)	<0.0001	32 (97.0)	6 (5.2)	<0.0001
**Hearing disturbance, n (%)**	2 (1.4)	16 (1.9)	ns	0	2 (1.8)	ns
**Cognitive impairment, n (%)**	23 (15.5)	13 (1.5)	<0.0001	12 (36.4)	11 (9.6)	<0.0001
**Sleeping disturbance, n (%)**	4 (2.7)	20 (2.4)	ns	0	4 (3.5)	ns
**Emotional instability, n (%)**	8 (5.4)	20 (2.4)	0.04	0	8 (7.0)	ns

E–encephalitis, ME–meningoencephalitis, ICU–intensive care unit, p_1_ –severe vs. non-severe cases, p_2_ –myelitis versus severe meningoencephalitis, ns–not significant.

The mean length of hospital stay was 12.0 ±6.5 days (min 1 day–max 129 days, n = 1000). A total of 298/1000 (29.8%) patients were treated in the intensive care unit (ICU). The mean treatment duration in the ICU was 3.8±10.0 (min <1 –max 127 days). Severe patients were treated in the hospital longer than non-severe patients (Table 2).

A total of 810/1000 (81%) patients presented sequelae on discharge. The most severe sequelae were observed among myelitic patients (Table 2).

A total of 7 patients died, 4 of them during the acute illness phase. There were 5/36 (14.9%) deaths in the myelitic group vs. 2/116 (1.7%) in severe ME/E, p = 0.009.

An autopsy was carried out on one fatal case. The 44-year-old previously healthy man died on the 5th day after the onset of the illness. He presented a double peak of fever up to 40˚C, meningeal symptoms, cerebellar ataxia, and dysarthria. The patient’s condition was improving. He had no complaints on the evening before death. The patient was conscious, had no clinical signs of brain edema, no pareses. He died suddenly while sleeping. Histologic examination showed severe brain edema, abundant hyperemia with perivascular hemorrhages, pathologic lymphocytic and monocytic perivascular cuffing, focal neuronal degeneration and necrosis in the anterior horns of the cervical part of spinal cord, in medulla oblongata, pons, basal ganglia, cerebellum (focal degeneration of Purkinje neurons), and meninges. According to the pathologist, sudden death was caused by acute heart failure of central origin.

### Predictors for severe course of the disease

The multivariate logistic analysis confirmed that a 1-year increase in the patient’s age increases the odds ratio for a severe course of the disease by 3%. The presence of comorbidities, high fever and protein concentration in CSF 1g/l and above doubles the odds ratio for severe TBE; the presence of meningeal signs increases it by 3 times. Delayed IgG production increases the odds ratio for severe TBE development by 5.3 times, the presence of abnormalities in CT by 6.8 times. Very similar predictors were associated with the evolution of severe ME/E form (Table 3). Univariate logistic regression showed that older age, CNS diseases, absence of meningeal signs, presence of bulbar syndrome, especially the presence of dysphagia, pleocytosis more than 500x10^6^/l in CSF, and delayed production of IgG predicted the development of myelitis in severe cases of TBE. After the completion of multivariate analysis, bulbar syndrome and absence of meningeal signs remained statistically significant predictors for myelitis (Table 3). Gender, hospitalization timeliness, ICU hospitalization time, and onset of qualitative or quantitative disturbances of consciousness did not show predictive abilities for severe TBE or the development of myelitis.

**Table 3:** Predictors for severe Tick-borne encephalitis.

Predictors for severe disease course (severe vs. non-severe)		
Covariate	Univariate analysis OR (95% CI); p	Multivariate analysis OR (95% CI); p
Age	1.03 (1.01–1.04); <0.0001	1.03 (1.01–1.04); 0.005
Comorbidities	1.82 (1.29–2.58); 0.001	2.08 (1.20–3.62); 0.009
Diabetes	ns	ns
Monophasic course	2.53 (1.78–3.60); <0.0001	1.64 (0.99–2.71); 0.054
Fever ≥ 40˚C	1.85 (1.17–2.92); 0.009	1.96 (1.05–3.65); 0.035
Meningeal signs	2.65 (1.75–4.00); <0.0001	2.97 (1.72–5.12); <0.0001
CRP ≥ 30 mg/l	2.56 (1.50–4.36); 0.001	ns
Pleocytosis ≥ 500x10^6^/l	2.75 (1.22–6.19); 0.015	ns
Neutrophils % in CSF	1.02 (1.01–1.03); <0.0001	1.02 (1.01–1.03); <0.0001
Protein ≥ 1g/l in CSF	2.22 (1.54–3.21); <0.0001	2.04 (1.19–3.51); 0.009
Delayed immune response of EEV IgG	3.20 (1.81–5.69); <0.0001	5.3 (2.22–12.7); <0.0001
Pathological findings in CT	4.65 (2.07–10.44); <0.0001	6.82 (1.6–29.17); 0.01
Predictors for myelitic form (myelitis vs. severe ME/E)		
Covariate	Univariate analysis OR (95% CI); p	Multivariate analysis OR (95% CI); p
Age	1.02 (1.00–1.05); 0.052	ns
Infected in living area	2.44 (1.00–5.99); 0.050	ns
CNS diseases	6.08 (1.38–26.84); 0.017	ns
Meningeal signs	0.29 (0.13–0.67); 0.004	0.01 (0.00–0.26); 0.008
Bulbar syndrome	2.77 (1.26–6.10); 0.011	14.86 (1.03–183.03); 0.035
Dysphagia	12.56 (3.18–49.53); <0.0001	-
Pleocytosis ≥ 500 x10^6^/l	4.52 (1.14–17.84); 0.031	ns
Delayed immune response of EEV IgG	4.04 (1.52–10.72); 0.005	ns
Predictors for severe ME/E form (severe ME/E vs. non-severe ME/E)		
Covariate	Univariate analysis OR (95% CI); p	Multivariate analysis OR (95% CI); p
Age	1.02 (1.00–1.03); 0.019	ns
Comorbidities	1.47 (0.99–2.17); 0.058	1.81 (0.99–3.29); 0.054
Monophasic course	2.12 (1.43–3.15); <0.0001	ns
Fever ≥ 40˚C	2.12 (1.29–3.48); 0.003	2.24 (1.15–4.36); 0.018
Meningeal signs	3.82 (2.26–6.44); <0.0001	3.38 (2.00–7.22); <0.0001
CRP ≥ 30 mg/l	2.64 (1.46–4.80); 0.001	ns
Neutrophils % in CSF	1.02 (1.01–1.02); <0.0001	1.02 (1.01–1.03); 0.001
Protein ≥ 1g/l in CSF	1.90 (1.26–2.88); 0.002	1.83 (1.01–3.30); 0.045
Delayed immune response of EEV IgG	2.11 (1.01–4.42); 0.048	4.11 (1.54–10.93); 0.005
Pathological findings in CT	4.98 (1.96–12.65); 0.001	8.15 (1.28–51.90); 0.026

ns–not significant.

## Discussion

TBE is a disease of substantial public health importance. With increasing intercontinental travel over the last decades, *flavivirus* infections such as TBE are posing a growing global health threat [16, 17]. Lithuania is a highly endemic country for TBE. There were 709 cases of illness and 5 deaths registered in 2019 [18]. In our study, the cases of TBE doubled in 2009 compared with the previous years 2005–2008, coinciding with an increase of TBE incidence in Lithuania. With regard to all TBE cases registered in Lithuania, the proportion of patients treated in the institutions participating in the study has increased since 2011: it constituted from 20% to 27% of the total TBE cases registered in Lithuania between 2011 and 2017, compared to 9% to 16% in the period between 2005 and 2010. According to our data, the proportion of severe cases is not associated with an increase in morbidity evaluating both annual morbidity dynamics and seasonal patterns. The peak of morbidity was in the 2nd half of the summer and early autumn, but the percentage of serious cases was the highest in June. It is difficult to find an explanation for the lack of association based on our study only. More detailed epidemiological studies are needed to clarify the seasonal nature and other epidemiological factors of severe forms of TBE. A better understanding of the complex epidemiological cycle of TBEV is necessary for the identification, monitoring and control of this virus [19].

The proportion of severe cases (14.6%) in our study was comparable with the data from neighboring Latvia (14.1%) [10], higher than in Poland (7.6%) [11], but lower than in Slovenia (68%) [13]. The high proportion of severe cases in Slovenia could be explained by study definitions. Not all cases of meningoencephalitis met the criteria for severe TBE in our study.

As is shown in recent studies, older age is a very important risk factor for severe TBE [13, 14]. In our study, patients with severe cases were older compared to those with non-severe TBE (mean age 55 years vs. 49 years, p<0.0001). The results of univariate and multivariate logistic regression showed that each additional 10 years increase the risk of severe TBE by 30%. Also, myelitic patients were older compared with severe ME/E patients mean age 60 years vs. 54 years (p 0.05). Although the logistic regression analysis did not reveal age as a statistically significant predictor for myelitis among patients with severe TBE, our study suggests that the risk of developing myelitis in the elderly is higher. Perhaps the relatively small number of myelitis forms influenced the results of the logistic regression. The risk of severe ME/E increases with age, and the risk of extremely severe myelitis is aggravated by the age of 60. In our study, as in Bogovich et al. [13], but unlike in Lenhard et al. [14], male sex was not a risk factor for severe disease. The majority of patients were infected by infected ticks, with only a small percentage of patients (7%) infected through milk, which was not related to the severity of the disease. It is important to note that 46% of patients became infected in their living area in the country and were not vaccinated. However, among myelitis patients, as many as 69% were infected in their living area (p = 0.05). In Lithuania, older people with low incomes tend to live in rural areas. This should be taken into account for the organization of publicly supported vaccination against TBE.

As in previous studies, one of the most common neurological signs of TBE was cerebellar ataxia [10–12]. This can be explained by the affinity of TBEV for Purkinje cells. The most extensive area of meningitis is around the cerebellum [12]. Ataxia was unrelated to the severe course of the disease in our study.

The most serious clinical form of TBE was myelitis, resulting in prolonged hospitalization, severe residual events, and death. Although the fact that the proportion of myelitis was lower than in other studies, 3.6% compared with 10% [12], 14.4% [14], the social and economic damage to the society was obvious. It is interesting to note that myelitic patients had headaches and meningeal signs less frequently compared with severe ME/E patients. Perhaps their condition was so severe that they did not notice the pain. Quantitative consciousness impairment and dysphasia were more common in severe ME/E than in myelitis. These are signs of higher-order brain dysfunction, and in the case of myelitis, the lesions predominate in the spinal cord and brain stem. In contrast to the previous studies, we classified meningoencephalitic/encephalitic forms as severe and non-severe (moderate and mild). Extrapyramidal tremor and parkinsonism were more common in non-severe ME/E than in the severe ME/E group. This indicates that lesions of the extrapyramidal nuclei are not related to the worst outcome, but are associated with moderate sequelae.

The lethality in our study was 0.7%, which is similar to some Latvian, Polish, and German studies [10–12]. In Europe, the overall case fatality ratio was 0.5% in the years 2012–2016 [20]. In contrast to the Lenhard et al. study [14], not all who died presented myelitis. One patient who presented severe ME/E died in the rehabilitation period of pneumonia. The problem is that the lethality of TBE can be underestimated because causes of death in the subacute period are attributed to pneumonia or other complications rather than TBE. Our study confirms the fact that the disease is potentially life-threatening [10, 11, 14, 21]. Not only those who present a coma or paresis, or those who are older may die. Dysfunction of the autonomic nervous system (ANS) is a potentially life-threatening situation. The tegmentum of the medulla and the pons, including raphe nuclei and the locus coerulus, i.e. the regions relevant to the ANS, were infected in over 50% of fatal cases [22]. Pathological studies from human post mortem CNS tissue revealed that TBEV selectively affects neurons in the brainstem, cerebellum, basal ganglia, and spinal cord. TBEV antigens were found in >50% of fatal cases in the medullar tegmentum and the pons, including its raphe nuclei and the locus coerulus, which are parts of the central ANS [23].

Recent studies have shown several clinical and laboratory parameters such as monophasic presentation [12, 13], underlying illness [13], CRP more than 30mg/l [13], delayed immune response of TBEV IgG [12], protein more than 1g/l in CSF and pathological findings in CT [11] to be associated with the severity of TBE. In our study, comorbidities, monophasic course, CRP more than 30mg/l, pleocytosis more than 500x10^6^/l, protein more than 1g/l in CSF, delayed immune response of IgG, and pathological findings in CT were predictors of severe disease. We did not find that blood leucocytosis is a predictor for severe disease as did Bogovič et al. [13]. Our data of logistic regression suggest that a high fever of more than 40˚C and signs of irritation of the meninges are associated with severe disease. This was not investigated in previous studies. Why do some patients develop severe myelitis, while others develop severe meningoencephalitis? Why do some patients develop severe ME/E and others non-severe? Can it be explained solely based on age or genetic factors? Older age is associated with immunosuppression. On the other hand, high fever, increased CRP, and high pleocytosis are markers of strong immune response, which can be caused by highly virulent strains of virus. We believe that the neuropathogenicity and the virulence of the virus may also have an effect on the course of the disease. Infection of any subtype is serious, but TBEV-Sib and TBEV-FE cause a more severe disease. The fatality rate of TBE caused by TBEV-Sib is about 20%, compared with 1–2% for TBEV-EU [24]. Also, TBE-Sib can cause chronic disease in 1.7% of cases [24]. TBEV-FE is associated with high rates of neurological sequelae, and up to 40% of cases are fatal [25]. Many aspects of TBEV biology remain unknown, and the virulence factors responsible for the different TBEV subtype pathologies have not yet been examined [25]. Although Lithuania is an endemic country for TBE and all three virus subtypes have been detected in the neighboring countries, no studies have been carried out yet to determine the virus subtypes.

## Conclusions

Our data from a very endemic region in eastern Lithuania show that although the proportion of severe cases is not associated with annual and seasonal increases in morbidity, Tick-borne encephalitis poses a growing health issue in Lithuania. A total of 15% of patients with TBE have a severe course of illness. About 70% of patients with myelitis, the most severe form of TBE, are infected in their living area. The prognostic factors for severe disease are older age, comorbidities, the most common of them arterial hypertension, monophasic course, a fever of 40˚C and above, CRP more than 30 mg/l, protein in CSF more than 1 g/l, delayed immune response of IgG, and pathological findings in CT such as brain edema, signs of intracranial hypertension (ventricle enlargement and tortuosity of the optic nerves), and white and gray matter hypodensities in temporal and frontal regions. These factors are also associated with the severe meningoencephalitic form. Age above 60 years, CNS disease, bulbar syndrome, pleocytosis 500x10^6^/l and above, and delayed immune response of TBEV IgG are predictors of the most severe myelitic form with poor outcome, and every patient with these factors has to be treated in an intensive care unit. Since Tick-borne encephalitis is a potentially life-threatening disease, every person living in a highly endemic country, as well as traveling to such countries, should be vaccinated against Tick-borne encephalitis.

## Supporting information

S1 Appendix Data file. (XLSX)
